The article "Computational and Mathematical Methods in Medicine Glioma Brain Tumor Detection and Classification Using Convolutional Neural Network" was published in 2022. Journal: Comput Math Methods Med.

# Computational and Mathematical Methods in Medicine Glioma Brain Tumor Detection and Classification Using Convolutional Neural Network

**DOI:** 10.1155/2022/4380901

**Published:** 2022-10-14

**Authors:** S. Saravanan, V. Vinoth Kumar, Velliangiri Sarveshwaran, Alagiri Indirajithu, D. Elangovan, Shaikh Muhammad Allayear

**Affiliations:** ^1^Department of Computer Science and Engineering, Vel Tech Rangarajan Dr. Sagunthala R&D Institute of Science and Technology, Avadi, Chennai, India; ^2^Department of Computer Science and Engineering, Jain (Deemed to Be University), Bangalore, India; ^3^Department of Computational Intelligence, SRM Institute of Science and Technology, Kattankulathur Campus, Chennai, India; ^4^School of Information Technology and Engineering, Vellore Institute of Technology, Vellore, 632014 Tamil Nadu, India; ^5^Department of Computer Science and Engineering, Panimalar Engineering College, Chennai, Tamil Nadu, India; ^6^Department of Multimedia and Creative Technology, Daffodil International University, Daffodil Smart City, Khagan, Ashulia, Dhaka, Bangladesh

## Abstract

The classification of the brain tumor image is playing a vital role in the medical image domain, and it directly assists the clinicians to understand the severity and to take an appropriate solution. The magnetic resonance imaging tool is used to analyze the brain tissues and to examine the different portion of brain circumstance. We propose the convolutional neural network database learning along with neighboring network limitation (CD_B_LNL) technique for brain tumor image classification in medical image processing domain. The proposed system architecture is constructed with multilayer-based metadata learning, and they have integrated with CNN layer to deliver the accurate information. The metadata-based vector encoding is used, and the type of coding estimation for extra dimension is known as sparse. In order to maintain the supervised data in terms of geometric format, the atoms of neighboring limitation are built based on a well-structured *k*-neighbored network. The resultant of the proposed system is considerably strong and subjective for classification. The proposed system used two different datasets, such as BRATS and REMBRANDT, and the proposed brain MRI classification technique outcome is more efficient than the other existing techniques.

## 1. Introduction

The term brain tumor is referred to as accumulation or rapid development of cells in the brain region. However, addressing the tumor location in the brain region is not as much as easier for radiologists. Basically, CT or MRI images can be used to identify the tumor portion from the brain region. A biopsy is a preamble clinical test used for brain cell extraction which can be done before the cerebrum surgery. The accurate measurement of a tumor cell or diagnosis is much needed without any technical or qualitative mistakes, whereas the advancement in machine learning may assist the radiologist of providing accurate information about the disease status [1, 2]. A CNN-based machine learning approach has been producing substantial outcomes in image classification and segmentation. Basically, there are three different types of brain tumors that have been classified by the CNN system approach. This CNN system or architecture has been tested with various existing system architectures, and the testing procedures involved T1-weighted contrast which improved MRI, and it is very simpler than the conventional models [3]. Four perspectives have been utilized to measure the system performance such as a grouping of 2-10-fold cross-examination technique, and it has 2 datasets. The defined system quality and capability have been tested by accepting one of the folding techniques, and the cross-examination of the subject portion was examined by involving the static image database called augmented framework. The designed framework outcome was 96.57% of accuracy, and it was the finest outcome when compared with other framework outcomes [4, 5]. The initial level of brain tumor examination can be executed with the help of a biopsy analysis report. However, this report is not up to the mark where the clinicians are not able to conclude the disease status history since it has a computational error and high time consumption. This demerit can be chased in order to utilize the deep learning technique in terms of performing multilevel classification of cerebrum tumor images [6]. This proposed system is being used to address the cerebrum tumor portion as quickly as anything without any technical flaws by using the CNN approach. This proposed system has three CNN architectures and classifications. However, the anticipation of the first CNN framework accuracy outcome is nearly about 99.34%, and the second model has five different types of cerebrum tumors such as benign, malignant, meningioma, metastatic, and pituitary, along with the obtained precision outcome of 92.67% [7]. The method describes the brain tumors are categorized into three grades (G) based on their characteristics such as GII, GIII, and GIV which obtained an accuracy rate of 98.15%. However, the specified CNN hyperlevel parameters are systematically routed by applying an optimized algorithm called “grid” [8]. Apparently, all these parameters are tuned with their respective characteristics by the proposed multilevel classification framework. The proposed system outcomes are compared with various traditional techniques like GoogleNET, ResNet50, and AlexNet [9].

The brain can be tested by various imaging modality, and the tested brain image is obtained from MRI or CT. However, while addressing the image parameter, quality, and image perception, the MRI achieved a better outcome than a CT image. The basic requirement of image analysis by the radiologist is nothing but time-consuming [10]. Low-level time consumption for image analysis for the radiologist is very essential while addressing the issue, and it may have chances of increasing the life span of the victim. The proposed framework uses CNN for image analysis and classification operation [11]. These CNN-based classified images are important for clinicians to obtain higher precision and accuracy values. However, this framework is referred to as a low complexity system, and it has five various types of brain MR images to produce an accurate analysis report [12]. The outcome of this proposed framework achieved 99.45% of the average value of the *F*1 score. However, the proposed system accuracy outcome was compared with existing framework techniques, and it obtained nearly about 99.69% of accuracy rate, which is a better score in their segment [13]. The MRI-based planes like sagittal, axial, and coronal are involved in training and testing the proposed framework in order to classify the brain malignant image [14, 15]. The two datasets have been used and belong to glioma-classified examination, and the resultant of the proposed system achieved the higher accuracy rate of 86.54% (IDH-mutation) and 90.8% (high/low glioma grades) [16]. Here, the graph-based semiadministrated learning technique has been used to evaluate the nonlabeled data labels which are presented in the dataset of the training mode, and it has an outcome that is slightly improved in performance which is found in a dataset of the testing mode [17, 18]. This method may overcome the data label missing issue in the dataset, and it really matters to the real-time scenario. To increase the performance of the dataset of the testing mode, an augmented dataset like GAN can be added in the dataset of the testing to enhance the overall system performance [19]. The testing of brain tumor multimodal MRI images has been done by deep learning technique from multiple-investigation analysis. This proposed system investigation examination has three different tumor sections such as classification, segmentation, and prediction (survival) [20]. The method of context-aware is with deep learning for segmentation (tumor) since it has the universal feature of context encoding technique. Further, this tumor image is involved in the classification scheme by applying the 3-dimensional convolutional neural network method [21].

The main focus of this framework is to highlight the classification scheme for MRI images of the brain tumor. This classification scheme is compatible with CNN, and it can address the images by utilizing the Keras dataset to create or manipulate the computerized CNN [22, 23]. The MRI images are segmented and extracted which can be done by preprocessing stage. The system proposes the novel classification scheme where the edge of the image can be identified by the edge detection method, and the ROI of the image has to be addressed and customized [24]. The data rate can be increased in training mode by utilizing an augmentation scheme. The resultant of the proposed system illustrates the smaller dataset is sophisticated to obtain a good accuracy, whereas we used to compare our results with some of the existing techniques like ResNet-50 and VGG-16 models [25]. This effort has focused on detecting the DDoS attack by emerging the deep learning-based classifier. The provision appeal from the users is composed and gathered as the record material. From the record file, some significant structures are designated for the organization by means of the Bhattacharya distance portion to diminish the training period of the classifier [26, 27]. Brain tumor happens due to unrestrained and fast development of cells. If not preserved at an early stage, it may lead to decease. Despite numerous important efforts and promising consequences in this area, precise division and classification continue a stimulating mission [28, 29]. A main contest for brain tumor recognition rises from the differences in tumor region, outline, and dimensions. The impartial of this review is to bring a complete literature on brain tumor discovery through magnetic resonance imagery to assist the researchers [30]. This survey enclosed the structure of brain tumors, openly obtainable datasets, improvement methods, division, feature removal, organization, and deep learning, transfer learning, and quantum machine learning for brain tumor examination. Lastly, this review delivers all significant works for the discovery of brain tumors with their advantages, boundaries, growths, and upcoming trends [31]. Medical histories in specific appear to be the consistent victims of hackers, and there are numerous information breach events throughout the history which have warranted the development of security procedures in contradiction of these threats, even though numerous security measures like cryptography, firewalls, and VPN are the combination of these methods that are essential for extreme security in medical image domain and data sharing.

## 2. Proposed System

### 2.1. Convolutional Neural Network Database Learning along with Neighboring Network

We proposed a fully systematic technique to classify the MR brain image, to support the clinicians to make or stick with the correct decision. However, making an accurate decision is not possible at a first sight or minimal amount of images. Here, the biased feature image representation has to be captured from brain MRI, in order to get the enhanced feature representation. The proposed convolutional neural network database learning along with the neighboring network limitation (CD_B_LNL) technique is used to anticipate the sparse mode feature illustration along with neighboring limitations for the respective layer. This neighboring limitation term can be utilized in order to maintain the neighboring data by implementing the manifold construction. CD_B_LNL system has different types of convolution network structures such as SoftMax and GoogleNET models.  Figure 1 represents the proposed system architecture, and it has four enlightening features such as (a) CD_B_LNL learns about feature illustration of a convolutional database for multilayer structure, and this illustration is encoded in a nonlinear plane; hence, this plane data can be employed. (b) This new plane or portion has to be addressed by a vector encoded-based multiple-layer database. If the addressed plane seems to be nonlinear, then the vector coding is known as sparse. Substantially, the unnecessary data can be removed while we implement the vector coding on biased information in order to obtain the estimated result. Let us consider, in our proposed framework, that executing the vector coding on solitary layer database learning can be customized only if it is a nonlinear mode; further, it can be changed as a linear-customized mode as per the system direction. (c) Let us consider the two-way operations like Laplacian graphical illustration, and supervised data seem to be well biased while using learned vector coding. The response received from the end layer shows that the learned vector coding can be preserved by Laplacian graphical illustration model. (d) This proposed CD_B_LNL framework executed the outcomes based on the two brain image datasets which are publicly available.

The performance outcome analysis of CD_B_LNL can be measured by five parameters such as precision, accuracy, recollect, stability loss, and *F*1 score.

Figure 1 applies the dataset inputs, and then, CNN framework is used to construct the neural network with the help of pooling. The output of pooling is associated with a fully connected CNN layer (cumulative input data). The consolidated output is connected with designed database-1 and needs to repeat the process in order to obtain the expected outcome like glioma and meningioma.

### 2.2. Datasets Used in CD_B_LNL

The proposed system uses two different types of datasets like BraTS and REMBRANDT. The dataset of BRATS (Multimodal Brain Tumor Image Segmentation Benchmark) is provided [13]. The brain MRI image dataset BraTS has been utilized in order to obtain the expected outcome of this proposed framework. The BraTS dataset is a dataset for brain tumor image segmentation. It has various grades of tumor images like benign, malignant, and pituitary.

It consists of 220 high-grade gliomas (HGG) and 54 low-grade gliomas (LGG) MRIs. The four MRI modalities are T1, T1c, T2, and T2FLAIR. Segmented “ground truth” provides about four intratumoral classes, viz., edema, enhancing tumor, nonenhancing tumor, and necrosis. Second, the proposed system uses the REMBRANDT database, and it has a cumulative amount of presurgical images which has multiple sequences of MR images. This database contains more than 110,000 images, especially for experimental purposes. Here, 135 patients' histories are taken based on the severity and brain tumor grade. This database contains oligodendrogliomas (OLI), ependymomas (EPY), carcinomatous meningitis (CAM), and some anonymous brain tumor categories. The database provides digitized images with 256 × 256-pixel resolution.  Figure 2 represents the BraTS dataset sample images for benign, malignant, and pituitary tumors.  Figure 3 illustrates the REMBRANDT database images for oligodendrogliomas (OLI), ependymomas (EPY), and carcinomatous meningitis (CAM) tumors [14].

### 2.3. Training the Database

However, training the database (metadata) is much essential to pick the correct image from the dataset; also, it is based on the image representation and characteristics. Let us consider the *Z* = [*a*_1_, *a*_2_, *a*_3_, ⋯.*a*_*n*_] ∈ *Q*^*c*∗*N*^ as a label of training image, and *B* ∈ *R*^*K*∗*N*^ is referred as sparse code of vector matrix. The database learning is represented as *D*_*B*_ ∈ *S*^*c*∗*K*^. However, the illustration of the nonlinear equation is  *CB* ≈ *Z*. Here, the database *D*_*B*_ may be learned like

(1) $$\begin{array}{c} \underset{D_{B},B}{\min}{\left\|Z-D_{B}B\right\|}_{F}^{2}+⋋\Theta \left(Z\right), \end{array}$$

(2) $$\begin{array}{c} \text{i}.\text{e }{\left\|d_{b}\right\|}_{2}^{2}\leq 1,\forall_{i}. \end{array}$$

Here, the error modification is representing as first term, and the coding limitation of the vector is declared as Θ(*Z*). However, this coding limitation can be represented in the form of Frobenius condition such as *l*_0_, *l*_1_, *l*_2_ ⋯ *l*_*n*_. The vector sparsity is being controlled by the positive scalar such as “⋋,” then the model complexity can be maintained or controlled by ‖*d*_*b*_‖_2_^2^ ≤ 1 condition. The main motive of this operation is to stop the *D*_*B*_ which is being literally huge; in outcome, it has very small values for “*Z*” (coding matrix). However, the notified parameters like *D*_*B*_ and *Z* can be optimized with the help of iteration modification towards convergence. The outcome of Equation (1) can achieve a better efficiency in terms of remodification operation, and it is being used for text or data mining with few classification features. Equation (1) is referred as unsupervised learning model; hence, it may consider to hold various type of noise functions in order to provide the information, then the supervised learning of this model can be illustrated as

(3) $$\begin{array}{c} \underset{\theta ,D_{B}}{\min}\underset{a\varepsilon Z}{\sum }R\left(l_{x},c_{x,}D_{B},\theta \right), \end{array}$$

(4) $$\begin{array}{c} ∴c_{x}=\text{argmin}{\left\|l_{x}-D_{B}c\right\|}_{2}^{2}+⋋\Theta \left(c\right). \end{array}$$

Here,

*l*_*x*_:Class label of “*x*”

*R*:Noise function

*θ*:Classification task (critical).

The parameters *D*_*B*_ and *θ* are to make the system biased capacity along with low cost of classifications. Hence, to achieve the optimized outcome of Equation (3), the methods like orthogonal matching pursuit and gradient allocation method can be utilized. Further, the outcome of Equation (3) will be an optimized outcome for *D*_*B*_.

### 2.4. CNN Database Learning (CND_B_L)

The proposed system framework is an extended work for existing database learning model from [12]. The main purpose of this proposed system is used to increase the capability of biased function and its features. This system must have a continuous flow of learning to follow the chronological order of CNN. Here, the filter convolution for CNN aggregates to make a flow in multiple layer convolutional databases by its sparse coding method. Here, the function of {*D*_*B*_}_*m*__*m*=1_^*M*^ is a convolutional database, where (*D*_*B*_)_*m*_*ε* *θ*^*d*_*b*_∗*K*_*m*_^ is the learning database and *K*_*m*_ is referred as the (*D*_*B*_)_*m*_ in size. Here, the “*Z*” is the convolutional illustration, and it can be written as

(5) $$\begin{array}{c} Z\approx {\left(D_{B}\right)}_{1}{\left(D_{B}\right)}_{2}{\left(D_{B}\right)}_{3}{\left(D_{B}\right)}_{4}\cdots ..{\left(D_{B}\right)}_{M}B_{M}. \end{array}$$

However, the neighboring limit has a decomposition, and it may be expressed as

(6) $$\begin{array}{c} {\left(D_{B}\right)}_{m-1}={\left(D_{B}\right)}_{M}B_{M}, \end{array}$$

(7) $$\begin{array}{c} Z={\left(D_{B}\right)}_{1}B_{1}, \end{array}$$

(8) $$\begin{array}{c} Z={\left(D_{B}\right)}_{1}{\left(D_{B}\right)}_{2}B_{2}, \end{array}$$

(9) $$\begin{array}{c} Z={\left(D_{B}\right)}_{1}{\left(D_{B}\right)}_{2}{\left(D_{B}\right)}_{3}B_{3}, \end{array}$$

(10) $$\begin{array}{c} Z={\left(D_{B}\right)}_{1}{\left(D_{B}\right)}_{2}{\left(D_{B}\right)}_{3}{\left(D_{B}\right)}_{4}B_{4}, \end{array}$$

(11) $$\begin{array}{c} Z={\left(D_{B}\right)}_{1}{\left(D_{B}\right)}_{2}{\left(D_{B}\right)}_{3}{\left(D_{B}\right)}_{4}{\left(D_{B}\right)}_{5}B_{5}, \end{array}$$

(12) $$\begin{array}{c} ∴Z={\left(D_{B}\right)}_{1}{\left(D_{B}\right)}_{2}\cdots ..{\left(D_{B}\right)}_{M}B_{M}. \end{array}$$

Equation (12) is a convolutional database learning, and the value of *B*_*M*_ is given as

(13) $$\begin{array}{c} B_{M}\epsilon Q^{N*K_{m}}. \end{array}$$

Hence, Equation (13) is referred as a vector coding matrix for the given system.

### 2.5. Different Stages of CD_B_LNL

This convolutional neural network database learning with neighboring limitation model has three different stages as follows:

- Abstract model function
- CND_B_LNL optimization
- Brain MR image testing and examination

### 2.6. Abstract Model Function (AMF)

The continuation of Equation (5) is the multiple layer database framework alongside with *M* layers; then, the vector coding *B*_*m*_ is expressed as

(14) $$\begin{array}{c} B_{m}\approx \vartheta \left[{\left(D_{B}\right)}_{m+1}B_{m+1}\right]. \end{array}$$

Here,

*ϑ*:Nonlinear operation

R_e_LU:Activation operation of hyperbolic and sigmoid.

This system describes the nature of each layer and its behavior or characteristics which have to be preserved for database monitoring. The coding vector is used to create a new input for every upcoming layer. The preserved data is much essential for retrieval of original sample of existing layer. The retrieval of original sample can be expressed as

(15) $$\begin{array}{c} \left(R_{e}\right)\left({\left(D_{B}\right)}_{1},{\left(D_{B}\right)}_{2},{\left(D_{B}\right)}_{3},\cdots {\left(D_{B}\right)}_{M}B_{M}\right)={\left\|Z-{\left(D_{B}\right)}_{1}\emptyset {\left(D_{B}\right)}_{2}\emptyset \cdots \emptyset {\left(D_{B}\right)}_{M}B_{M}\right\|}_{F}^{2}+⋋\Theta \left({\text{B}}_{\text{M}}\right). \end{array}$$

Here, ⋋ is referred as parameter of organization, and the respective rank operator Θ(B_M_) is calculated as

(16) $$\begin{array}{c} B_{M}\approx S_{H},\\ ∴{\left\|B_{M}-S_{H}\right\|}_{F}^{2}, \end{array}$$

where

(17) $$\begin{array}{c} S\;\epsilon \;Q^{K_{m}*C}\&H\;\epsilon \;Q^{C*N}. \end{array}$$

*C* is the data sample class number.

In order to enhance this performance of classification, the neighboring data is playing the primary role in any type of database learning. Hence, the atoms found in database learning is very stable than original data. In this regard, the Laplacian hazard function is used to manifold the information. In this case, this proposed system utilizes a supervised scheme by its neighboring graph (*E*), when it comes to database (*D*_*B*_)*_m_* found in the existing layer. However, the portions of neighboring graph elements like *E*_*i*,*j*_ are described as

(18) $$\begin{array}{c} E_{i,j}=\left\{\begin{array}{cc} \exp\left[-\frac{{\left(\left\|{\left(d_{b}\right)}_{M,i}-{\left(d_{b}\right)}_{M,j}\right\|\right)}^{2}}{\sigma },\right. & \text{ if }{\left(d_{b}\right)}_{M,i}\epsilon \text{KNN}\left[{\left(d_{b}\right)}_{M,j}\right]\\ 0, & \text{else} \end{array}\right\}, \end{array}$$

where

*σ*:Flexible parameter.

Here, Equation (18) has to reconstruct with Laplacian regularization, then the equation can be expressed as

(19) $$\begin{array}{c} ∴{\left(R_{e}\right)}_{2}\left(B_{M}\right)=T_{r}\left(B_{M}^{T}*LB_{M}\right). \end{array}$$

Here, the Laplacian matrix “*L*” can be expressed as

(20) $$\begin{array}{c} L=\mathrm{diag}\left(E_{1},E_{2},E_{3},E_{4},\cdots \cdots E_{KM}\right)-E, \end{array}$$

where

(21) $$\begin{array}{c} E_{i}=\overset{K_{M}}{\underset{j=1}{\sum }}E_{i,j}. \end{array}$$

Further, Equation (21) can be used for biased database and utilize the Softmax classifier loss in the existing or final layer in the CNN model.

(22) $$\begin{array}{c} {\left(R_{e}\right)}_{3}\left(B_{m},\theta \right)=-\frac{1}{M}\overset{M}{\underset{i=1}{\sum }}\underset{C=1}{\sum }p_{c,i}\log\frac{e^{\theta_{C}^{T}{\left(d_{b}\right)}_{M,i}}}{\sum_{u=1}^{C}e^{\theta_{u}^{T}{\left(d_{b}\right)}_{M,i}}}. \end{array}$$

In Equation (22), the *p*_*c*,*i*_ may be the probability value of the label, and it can be expressed as *o*_*M*,*j*_, and its corresponding class is “*C*,” i.e., *θ* = [*θ*_1_, *θ*_2_, *θ*_3_, *θ*_4_ ⋯ .*θ*_*c*_). It is belonging to softmax layer, and it is flexible in operation. In the classification of a brain tumor image, it requires three basic ordinary functions, and it is denoted as (*R*_*e*_)_1_, (*R*_*e*_)_2_, and (*R*_*e*_)_3_. When we combine these three functions along with convolutional database learning with classifier, then the final equation of the CNN-based database learning model is expressed as

(23) $$\begin{array}{c} \text{argmin}{\left(R_{e}\right)}_{1}\left[{\left(D_{B}\right)}_{1},{\left(D_{B}\right)}_{2},{\left(D_{B}\right)}_{3},\cdots .{\left(D_{B}\right)}_{M},B_{M}\right]+{\left(R_{e}\right)}_{2}B_{M}+{\left(R_{e}\right)}_{3}\left(B_{M},\theta \right), \end{array}$$

(24) $$\begin{array}{c} \text{i}.\text{e}{\left\|{\left(d_{b}\right)}_{i}\right\|}_{2}^{2}\leq 1,\forall_{i}. \end{array}$$

From Equation (23), it clearly shows the decent improvement found in database learning during the optimization operation. However, the outcome of the model shows the stability of the classifier in terms of various potentials like biased and numerical values of database system coding.

### 2.7. CD_B_LNL Optimization

From Equation (23), it provides the decent level of improvements in database learning, though it is not up to the standard level. In this regard, we have to find the other alternate solution to obtain the desired outcome. So, we may take database values like [(*D*_*B*_)_1_, (*D*_*B*_)_2_, (*D*_*B*_)_3_, ⋯.(*D*_*B*_)_*M*_] along with matrix coding “*B*” (since it has a classifier ‘*θ*′). The step by step operation is required, and repetition in each step that is used to calculate the parameter needs to be fixed by another parameter. In order to fix this issue, the updating of the database is required, so the chain regulation is being used to calculate the database values in each layer {(*D*_*B*_)_*M*_(1 ≤ *m* ≤ *M*)}.

(25) $$\begin{array}{c} \frac{\partial \left(R_{e}\right)}{\partial {\left(D_{B}\right)}_{M}}=\frac{\partial \left(R_{e}\right)}{\partial \left({\left(D_{B}\right)}_{M}B_{M}\right)}B_{M}^{T}=\left[\frac{\partial \left(R_{e}\right)}{\partial \vartheta \left({\left(D_{B}\right)}_{M}B_{M}\right)}⨀\vartheta^{\prime }\left({\left(D_{B}\right)}_{M}B_{M}\right)\right]B_{M}^{T}=\left[\frac{\partial \left(R_{e}\right)}{\partial B_{\left(m-1\right)}}⨀\vartheta^{\prime }\left({\left(D_{B}\right)}_{M}B_{M}\right)\right]B_{M}^{T}. \end{array}$$

Here, ⨀ represents the multiplication for each element in database; once the database (*D*_*B*_)_*M*_ has been achieved, then Equation (18) can be applied in order to build the graph value of Laplacian regularization. The classifier which we used for classification of brain image is softmax layer, and the classifier optimization parameter can be calculated.

(26) $$\begin{array}{c} \frac{\partial \left(R_{e}\right)}{\partial \theta_{C}}=-\frac{1}{M}\overset{M}{\underset{i=1}{\sum }}\overset{C}{\underset{C=1}{\sum }}f_{C,i}\left(1-\frac{e^{\theta_{c}^{T}b_{M,i}}}{\sum_{u=1}^{C}e^{\theta_{c}^{T}b_{M,i}}}\right)\beta_{M,i}^{T}. \end{array}$$

Equation (26) is referred as convolutional database learning with neighboring network optimization equation.

### 2.8. Brain MR Image Testing and Examination

The descriptor of the feature can be denoted as “*y*,” and it is depending on the optimization outcome. It is expressed as, *U*, *K*, and *θ* for [(*D*_*B*_)_1_, (*D*_*B*_)_2_, (*D*_*B*_)_3_, ⋯.(*D*_*B*_)_*M*_].

Then, the calculation of the encoding of the database can be forms as

(27) $$\begin{array}{c} \underset{b_{M}}{\min}{\left\|y-{\left(D_{B}\right)}_{1}\vartheta \left({\left(D_{B}\right)}_{2}\vartheta {\left(D_{B}\right)}_{3}\vartheta \left(\cdots \vartheta \left({\left(D_{B}\right)}_{M}b_{M}\right)\right)\right)\right\|}_{F}^{2}+{⋋}_{2}{\left\|b_{M}-UK\right\|}_{F}^{2}. \end{array}$$

Further, the classification feature can be executed by softmax layer, then the probability of the label of “*y*” is finalized to class “*c*,” then the equation can be written as

(28) $$\begin{array}{c} g_{c=}\frac{e^{\theta_{v}^{T}b_{M}}}{\sum_{v=1}^{C}e^{\theta_{v}^{T}b_{M}}}. \end{array}$$

Equation (28) is referred as brain MRI image testing and examination equation for the proposed model.

## 3. Results and Discussions

### 3.1. Experimental Setup

In our proposed system, we may have 1200 images from the BraTS dataset and the entire REMBRANDT dataset utilized for simulation purposes. Here, the brain MR images are customized into 227 × 227 size in order to utilize the GoogLeNet. Let us consider that all layers in the CDBLNL, which may make use of 3 × 3 size filters. Here, the system requires the optimizer to optimize the model. So, we took stochastic gradient descent, and the Tensor-Flow is being used to make system implementation. However, the function is being activated by ReLU operation. The first and preamble step of the database starts from (*D*_*B*_)_1_ and *B*_1_. The function of K-SVD architecture is utilized in every class of information, and it may get integrated with subclass database into the main database  (*D*_*B*_); finally, the function of fully learned database and coding vector has been obtained from the existing layer of the model [(*D*_*B*_)_*M*_, *B*_*M*_]. The consolidated parameters like (⋋_1_, ⋋_2_, ⋋_3_) in CD_B_LNL may be used in grid control mode search {0.001, 0.01, 0.1, 1, 10, 100}. The comparable outcome of the model is obtained, and it has been validated by a fivefold cross-validation method. However, the training and testing fold values are validated, and it is being used 70% and 30%, respectively. In the proposed system, the function of this model is being executed in frequent intervals of time, and we took almost 10 values during the execution, and it has been summarized; then, the average value is being taken from the summarized value.

There are five parameters that have been taken to evaluate the proposed system performance such as precision, accuracy, recollect (recall), balance loss, and *F*1 score, respectively. A lot of techniques have been used to classify the tumor images from the brain region. However, we made a comparative analysis between conventional machine learning and deep learning for experimental intention. Most of the experiments in conventional ML technique used support vector machine (SVM) [15] along with RDF kernel to make the reliable structure, the database learning technique consistent label (KSVD) [2], and the coactive adaptive neural fuzzy expert system (CANFES) [8], and finally, CNN is designed to automatically and adaptively learn spatial hierarchies of features through back-propagation by using multiple building blocks [11]. During the experiment, the statistical texture features like mean, median, contrast, energy, and variance have been utilized, and comparison outcome of deep learning base KSVD features, and we derive the features from CNN model GoogLeNet and may execute these outcomes on KSVD2. The devices which we have used for our experimental purpose have an i5 Intel processor (10^th^ Gen) and 8 Gb of RAM. The programming language Python (along with Keras libraries and tensor flow) is used as a basic platform to execute any type of implementation techniques.

#### 3.1.1. Database Availability

The brain tumor image database used for experimental execution and analysis in our proposed framework are publicly available, and information is given.

- BraTS: https://www.smir.ch/BRATS/Start2015
- REMBRANDT: https://wiki.cancerimagingarchive.net/display/Public/REMBRANDT

### 3.2. BraTS Database Experimental Outcome: CD_B_LNL

The proposed system performance outcome of classification can be evaluated by BraTS dataset. This type of dataset contains three kinds of tumor images such as benign, malignant, and pituitary tumors.

Table 1 illustrates the BraTS dataset-based confusion matrix of CD_B_LNL model, and it clearly shows the pituitary has the maximum accuracy in the table, and the second highest accuracy goes to malignant tumors, and the least accuracy value goes to benign tumors. Further, Table 2 consists of various parameters like precision, recollect (recall), accuracy, stability loss, and *F*1 score to evaluate the process, and it has the average value of each parameters. The proposed system classification performance can be evaluated by tenfold model. Here, Table 2 illustrates the obtained parameter outcomes CD_B_LNL model, and it shows high average and small deviation value on accuracy. Then, the proposed system performance outcomes are compared with various existing techniques such as SVM_RBF, LC-KSVD1, LC-KSVD2, CANFES, and CNN, respectively.

Table 3 represents the proposed system performance metric comparison outcome with other traditional machine learning models. Table 3 has five parameters and tenfold metric outcomes, and these parameter outcomes are cumulatively summarized, and the average value of each model outcome is highlighted, respectively.  Figure 4 shows the graphical illustration of the performance metric comparison of proposed system outcome with existing model outcomes. From Table 3, the proposed system provides a better outcome in all parameters when compared with other traditional machine learning techniques. From the feature of deep learning architecture, the proposed system addresses the nonlinear portion indexes like encoding and feature representation for multiple layer database learning. The sparse code data can be preserved by Laplacian regularization for neighboring limitations in terms of enhancing the biased ability of the model. However, from the outcome of the proposed system, we may understand that the deep feature is well-adapted model for image categorization.

### 3.3. REMBRANDT Database Experimental Outcome: CD_B_LNL

The proposed CD_B_LNL system uses BraTS and REMBRANDT databases. Then, the performance classification metric outcome of CD_B_LNL is achieved from REMBRANDT database, and it contains three kinds of tumor image types like OLI, CPY, and CAM.

Table 4 illustrates the REMBRANDT dataset-based confusion matrix of CD_B_LNL model, and the classification rate of OLI is 0.9127, CPY is 0.9541, and CAM is 0.9310. Further, Table 5 shows various parameters such as precision, recollect (recall), accuracy, stability loss, and *F*1 score to evaluate the process, and it shows the average value of each parameters. The proposed system classification performance can be evaluated by tenfold model.

Here, Table 5 illustrates the obtained parameter outcomes CD_B_LNL model, and it shows high average and small deviation value on accuracy. Then, the proposed system performance outcomes are compared with various existing techniques such as SVM RBF, KSVD1, KSVD2, CANFES, and CNN, respectively.  Table 6 represents the proposed system performance metric comparison outcome with other traditional machine learning models.  Table 6 has five parameters and tenfold metric outcomes, and these parameter outcomes are cumulatively summarized, and the average value of each model outcome is highlighted, respectively.  Figure 5 shows the graphical illustration of the performance metric comparison of proposed system outcome with existing model outcomes. From Table 6, the proposed system provides a better outcome in all parameters when compared with other traditional machine learning techniques.

The proposed system classification performance outcomes based on BraTS and REMBRANDT database are shown in Table 7. The graphical representation of proposed CD_B_LNL classification performance outcomes on BraTS and REMBRANDT database is shown in Figure 6.

## 4. Parameter Index Evaluation

The proposed system parameter index sensitivity has been analyzed on both BraTS and REMBRANDT database. However, the consolidated parameters such as ⋋_1_, ⋋_2_, and⋋_3_ in CD_B_LNL can be used in grid control mode search {0.001…0.1…100}. Let us consider and assign the parameter values as per the grid search, then the assigned values are “*ω*_1_ = *ω*_2_” and the classification accuracy visualization of CD_B_LNL along with various data of *ω*_2_ = *ω*_3_, respectively.

### 4.1. Index Evaluation

When (⋋_1_ = ⋋_2_), the CD_B_LNL classification accuracy value has to be visualized with other parameters (⋋_2_and⋋_3_).

When (⋋_2_ = ⋋_3_), the classification accuracy value illustration is taken along with accompanied parameter values (⋋_1_and⋋_3_).

When (⋋_1_ = ⋋_3_), classification accuracy score visualization is based on other parameter values (⋋_1_and⋋_2_).

The proposed CD_B_LNL classification accuracy (parameter index examination) values on BraTS and REMBRANDT are shown in Figures 7 and 8. Let us imagine the “*G*” is the number of layers presented on both BraTS and REMBRANDT databases. Assume the grid value,

(29) $$\begin{array}{c} G=\left\{2.3,\cdots .8\right\}. \end{array}$$

From Equation (29), in order to examine the effect of CD_B_LNL classification accuracy, the grid value of accuracy is shown in Figure 8. However, the proposed system accuracy rate is improving when “*G*” value increases from 1 to 3. Then, when the grid value *G* > 3, then the proposed model classification accuracy is more reliable on both BraTS and REMBRANDT databases.

## 5. Conclusion

In order to classify the brain tumor MR images more quickly and precisely, we propose the CD_B_LNL model. The contribution of the convolutional neural network is much essential to search the nonlinear portion of sparse illustration. The various classes and their coding vectors provided the biased approximation information. However, the proposed method utilizes the neighboring limitation of atoms in order to maintain the structure code of manifold. The proposed system extracts the meaningful convolutional features systematically which is based on the deep learning architecture. The brain tumor classification types like benign, malignant, and pituitary on BraTS database and the OLI, CPY, and CAM images on RANBRANDT have been executed, and we obtained the high-performance value in all parameters like precision, recall accuracy, balance loss, and *F*1 score, respectively.

## Figures and Tables

**Figure 1:** (a) Proposed system block diagram; (b) proposed system CD_B_LNL architecture.

**Figure 2:** BraTS dataset sample brain MR images.

**Figure 3:** REMBRANDT dataset sample brain MR images.

**Figure 4:** BraTS database classification performance of CD_B_LNL.

**Figure 5:** REMBRANDT database classification performance of CD_B_LNL.

**Figure 6:** CD_B_LNL classification performance outcomes based on BraTS and REMBRANDT database.

**Figure 7:** Parameter index sensitivity of CD_B_LNL on BraTS database (a–c).

**Figure 8:** Parameter index sensitivity of CD_B_LNL on REMBRANDT database (a–c).

**Table 1:** BraTS dataset-based confusion matrix of CD_B_LNL model.

Types	Benign	Malignant	Pituitary
Benign	0.790	0.081	0.029
Malignant	0.039	0.899	0.0059
Pituitary	0.0089	0.0069	0.893

**Table 2:** BraTS dataset-based classification performance of CD_B_LNL model.

Manifold	Mode of operation	Precision	Recall	Accuracy	Stability loss	*F*1 score
I	Training	96.1	95.1	97.1	97.1	95.1
	Testing	95.2	95.6	97.3	96.9	95.2
II	Training	94.8	96.1	97.01	96.8	96.1
	Testing	95.01	95.3	97.03	96.9	95.3
III	Training	96.1	95.3	96.89	97.1	95.7
	Testing	94.9	95.1	97.4	97.1	95.9
IV	Training	95.3	96.1	97.2	96.9	95.9
	Testing	94.8	95.6	97.45	96.09	95.3
V	Training	95.6	96.2	97.8	97.01	96.1
	Testing	94.7	95.7	96.9	96.9	96.3
VI	Training	96.1	95.1	97.1	97.1	95.1
	Testing	95.2	95.6	97.2	96.9	95.2
VII	Training	94.8	96.11	97.08	96.8	96.1
	Testing	95.07	95.3	97.07	96.9	95.3
VIII	Training	96.1	95.32	96.82	97.1	95.7
	Testing	94.9	95.12	97.41	97.1	95.9
IX	Training	95.3	96.11	97.3	96.9	95.9
	Testing	94.79	95.63	97.44	96.09	95.3
X	Training	95.59	96.28	97.85	97.01	96.1
	Testing	94.74	95.74	96.89	96.9	96.8
Average (%)		95.255	95.6205	97.212	96.88	95.715

**Table 3:** Performance metric comparison of proposed system with existing techniques.

Parameters/models	SVM RBF	KSVD1	KSVD2	CANFES	CNN	CD_B_LNL
Precision	82.9	83.5	86.1	90.5	89.8	95.3
Recall	81.9	82.9	87.4	89.8	91.5	95.6
Accuracy	85.8	88.8	89.2	91.8	94.6	97.2
Balance loss	84.6	87.5	88.9	91.2	94.9	96.8
*F*1 score	85.1	89.1	88.95	91.1	90.9	95.7

**Table 4:** REMBRANDT dataset-based confusion matrix of CD_B_LNL model.

Types	OLI	CPY	CAM
OLI	0.0621	0.9127	0.0252
CPY	0.9541	0.0899	0.0590
CAM	0.0589	0.0069	0.9310

**Table 5:** REMBRANDT dataset-based classification performance of CD_B_LNL model.

Manifold	Mode of operation	Precision	Recall	Accuracy	Stability loss	*F*1 score
I	Training	95.81	93.94	97.94	95.91	94.54
	Testing	95.74	93.81	97.84	95.74	94.34
II	Training	95.74	93.89	97.91	95.89	94.56
	Testing	95.68	93.75	97.81	95.70	94.44
III	Training	95.71	93.91	97.93	95.86	94.38
	Testing	95.67	93.82	97.85	95.75	94.29
IV	Training	95.56	93.94	97.91	95.84	94.41
	Testing	95.49	93.86	97.83	95.71	94.36
V	Training	95.67	93.85	97.74	95.90	94.40
	Testing	95.57	93.78	97.69	95.86	94.35
VI	Training	95.55	93.86	97.78	95.81	94.28
	Testing	95.49	93.81	97.65	95.74	94.15
VII	Training	95.68	93.91	97.84	95.91	94.22
	Testing	95.58	93.87	97.78	95.88	94.19
VIII	Training	95.76	93.90	97.86	95.58	94.33
	Testing	95.69	93.82	97.79	95.47	94.28
IX	Training	95.80	93.92	97.80	95.77	94.37
	Testing	95.71	93.88	97.75	95.66	94.29
X	Training	95.77	93.87	97.88	95.74	94.33
	Testing	95.67	93.76	97.79	95.68	94.29
Average (%)		95.667	93.8575	97.8185	95.77	94.34

**Table 6:** Performance metric comparison of proposed system with existing techniques.

Parameters/models	SVM RBF	KSVD1	KSVD2	CANFES	CNN	CD_B_LNL
Precision	81.9	83.5	90.1	88.2	90.8	95.6
Recall	80.9	82.9	89.4	89.8	91.5	93.8
Accuracy	84.8	88.8	90.2	87.8	91.6	97.8
Balance loss	83.6	87.5	90.9	87.2	90.9	95.7
*F*1 score	84.1	89.1	89.95	88.1	90.1	94.3

**Table 7:** CD_B_LNL classification performance outcome on BraTS and REMBRANDT database.

Parameters/models	BraTS	REMBRANDT
Precision	95.3	95.6
Recall	95.6	93.8
Accuracy	97.2	97.8
Balance loss	96.8	95.7
*F*1 score	95.7	94.3

## Data Availability

The data used to support the findings of this study are included within the article.
